This article has been retracted.

# MicroRNA-302b suppresses cell proliferation by targeting EGFR in human hepatocellular carcinoma SMMC-7721 cells

**DOI:** 10.1186/1471-2407-13-448

**Published:** 2013-10-02

**Authors:** Lumin Wang, Jiayi Yao, Xin Shi, Lili Hu, Zongfang Li, Tusheng Song, Chen Huang

**Affiliations:** 1 Department of Genetics and Molecular Biology, Xi’an Jiaotong University Health Science Center, No.76 West Yanta Road, Xi’an, Shaanxi 710061, P.R. China; 2 Xi’an IV People’s Hospital, Xi’an, Shaanxi, P.R. China; 3 Engineering Research Center of Biotherapy and Translational Medicine of Shaanxi Province, Xi’an, Shaanxi, P.R. China; 4 Key Laboratory of Environment and Genes Related to Diseases, Xi’an Jiaotong University Health Science Center, Xi’an, Shaanxi, China; 5 Cardiovascular Research Center, Xi’an Jiaotong University Health Science Center, Xi’an, Shaanxi, P.R. China

**Keywords:** miR-302b, Hepatocellular carcinoma, EGFR, Proliferation, Cell cycle

## Abstract

**Background:**

MicroRNAs are regulators that can play an essential role in tumorigenesis. Although miR-302 families have been suggested to be tumor repressors in human cancer, the mechanism by which they suppress tumor development remains to be defined. In this study, we discover that miR302b suppresses tumor proliferation may due to directly targeting EGFR in human hepatocellular carcinoma (HCC).

**Methods:**

QRT-PCR was used to assess miR-302b and EGFR expression in 27 pairs of clinical hepatocellular carcinoma tissues and their corresponding adjacent nontumorous liver tissues. MTT, colony formation, immunofluorescence staining, and cell cycle assays were used to examine the tumor suppressor role of miR302b in cell proliferation. Luciferase assays were performed to assess the EGFR was a novel target of miR-302b. Western blot assay was used to validate the protein expression level.

**Results:**

We demonstrated that miR-302b was frequently down-regulated, whereas EGFR was up-regulated in 27 pairs of clinical HCC and non-tumorous counterparts. The dual-luciferase reporter assays revealed that EGFR was a novel target of miR-302b. Re-expression of miR-302b resulted in the inhibition of proliferation in hepatocellular carcinoma SMMC-7721 cells. The silencing of EGFR by miR-302b or siEGFR led to down-regulation of proliferation-related proteins, such as AKT2, CCND1, and CDK2.

**Conclusion:**

miR-302b suppresses HCC growth may due to targeting the EGFR/AKT2/CCND1 pathway.

## Background

Hepatocelluar carcinoma (HCC) is the third leading cause of cancer-related deaths worldwide, and the burden of this devastating cancer is expected to increase further in the coming years [1]. Due to the difficulty of effectively diagnosing HCC at its early stage, only about 10 to 20% of patients with hepatocellular carcinoma are currently eligible for surgical intervention [2-6]. Therefore, elucidating the molecular mechanisms involved in HCC is essential for developing cancer prevention strategies and possible guiding disease management in the clinic.

Accumulating evidence suggests that microRNAs (miRNAs) are involved in the initiation and progression of HCC [7]. First, the 22nt noncoding miRNAs act as key regulators of various fundamental biological processes, such as development, differentiation, apoptosis, and cell proliferation, in which common pathways are shared with cancer [8-11]. Second, bioinformation analyses estimate that miRNAs may regulate as much as 30% of the human protein coding genes, including oncogenes and tumor suppressors, suggesting that these small RNAs may act to coordinate the interplay between complex signal transduction pathways [12]. Third, increasing evidence shows that the expression of miRNAs is remarkably deregulated in cancer due to multiple epigenetic and genomic alterations. Fourth, several miRNAs themselves have been demonstrated to serve as tumor suppressor genes or oncogenes in tumors [13-15].

The miR-302 family consists of four highly-homologous miRNA members, which are transcribed together as a noncoding RNA cluster containing mir-302b, mir-302c, mir-302a, mir-302d, and mir-367 in a 5′-to-3′ direction [16]. To date, miR-302 s have been proven to post-transcriptionally regulate CCND1 and CDK4, therefore affecting cell cycle progression. Other studies have demonstrated the tumor suppressive activity of miR-302 in human pluripotent stem cell by both the CCNE-CDK2 and CCND-CDK4/6 pathways in G1-S cell cycle transition. Although miR-302 has been suggested to have tumor suppressor potential, the present studies focused on the self-renewal and proliferation properties of miR-302b in the stemness maintenance of embryonic stem cells (ESCs) or tumor stem cell properties in advanced cancer cells [17,18]. So, the relationship between miR-320b and cancers needs to be investigated further.

In this research, we analyzed the miR-302b targets by bioinformatics software, and found that miR-302b can target EGFR. Next, we found that miR-302b was frequently down-regulated in HCC tissues and cells. Further, in vitro experiments proved that the re-expression of miR-302b inhibited HCC proliferation dramatically, and arrested the HCC cell cycle at the G1/S phase. The dual-luciferase reporter assays further demonstrated that EGFR was a novel target of miR-302b. The silencing of EGFR by miR-302b or siEGFR led to the down-regulation of cell-cycle related proteins, such as AKT2, CCND1, and CDK2, strongly suggesting that miR-302b suppresses the growth of SMMC-7721 cells by targeting EGFR involved the EGFR/AKT2/CCND1 pathway.

## Methods

### Cell lines and tissue specimens

Bel7402, SMMC-7721, HepG2, Hep3B, and HL-7702 cells were maintained in 1640 medium (1640, PAA Laboratories GmbH, Pasching, Austria), supplemented with 10% fetal bovine serum (FBS, PAA Laboratories GmbH, Pasching, Austria). Cells were maintained at 37°C in a humidified chamber with 95% air and 5% CO_2_. 27 paired HCCs and adjacent non-tumor liver tissues were collected from patients undergoing resection of HCC at the Hepatobiliary Surgery Department of the First Affiliated Hospital of Xi’an Jiaotong University, P.R. China. No local or systemic treatment had been conducted before operation. Tissue samples were immediately snap frozen in liquid nitrogen until RNA extraction. Both tumor and non-tumor tissues were histologically confirmed. Informed consent was obtained from each patient and was approved by the Institute Research Ethics Committee at the Cancer Center, Xi’an Jiaotong University.

### Plasmid constructions

pcDNA™6.2-GW/EmGFP-miR vector (Invitrogen) was used to construct vectors of re-expression miR-302b. First, we inserted EcoRI and HindIII sites into the MCS of the vector. Then, the miR-302b was chemically synthesized and cloned into pcDNA™6.2-GW/EmGFP-miR vector between the EcoRI and HindIII sites. RegRNA (A Regulatory RNA Motifs and Elements Finder http://regrna.mbc.nctu.edu.tw/), TargetScan (http://www.targetscan.org/) and DIANA (http://diana.cslab.ece.ntua.gr/microT/) were used for gene-related specified microRNA prediction. Through bioinformatics analysis, we got the predicted fragment of targeted gene (EGFR), which was associated with miR302b. Specified fragments of EGFR were chemically synthesized, and are shown in supporting Table 1. The luciferase-UTR reporter constructions were generated by introducing the Wt/Mut-EGFR 3′-UTR, carrying a putative miR-302b binding site into pmirGLO Dual-Luciferase miRNA Target Expression vector (Promega) between the XhoI and SacI sites.

**Table 1:** Primers and oligonucleotides used in this work

**Name**	**Sequence (5′-3′)**
Pri-miR-302b-S	5′-AATTCGCTCCCTTCAACTTTAACATGGAAGTGCTTTCTGTGACTTTAAAAGTAAGTGCTTCCATGTTTTAGTAGGAGTA-3′
Pri-miR-302b-A	5′-AGCTTACTCCTACTAAAACATGGAAGCACTTACTTTTAAAGTCACAGAAAGCACTTCCATGTTAAAGTTGAAGGGAGCG-3′
EGFR 3′UTR-S	5′-CAAGAAGCTTGCTGGTAGCACTTGC- 3′
EGFR 3′UTR-A	5′-TCGAGCAAGTGCTACCAGCAAGCTTCTTGAGCT- 3′.
EGFR 3′UTR-MS	5′-CAAGAAGCTTGCTGGCAGCGTTTGC-3′
EGFR 3′UTR-MA	5′-TCGAGCAAACGCTGCCAGCAAGCTTCTTGAGCT-3′
siRNA-ctrl-S	5′-ACCGAACGTGTCACGT-3′
siRNA-ctrl-A	5′-ACGTGACACGTTCGGAGAATT-3′
siEGFR-S	5′-AACACAGTGGAGCGAATTCCT-3′
siEGFR-A	5′-AGGAATTCGCTCCACTGTGTT-3′
miR-302b RT	5′-TGCTTAAGTGCTTCCATGTT-3′
miR-302b-F	5′-ATCCAGTGCGTGTCGTG-3′
miR-302b-R	5′-TGCTTAAGTGCTTCCATGTT-3′
Inhibitor-ctrl	5′-TGACTGTACTGACTCGACTG-3′
MiR-302b inhibitor	5′ -TGATTTTGTACCTTCTGGAAT-3
EGFR-F	5′-GCCTTGACTGAGGACAGCA-3′
EGFR-R	5′-TTTGGGAACGGACTGGTTTA-3′
β-actin-F	5′-CGGGAAGCTTGTCATCAATGG-3′
β-actin-R	5′-GGCAGTGATGGCATGGACTG-3′
U6 RT	5′-GTCGTATCCAGTGCAGGGTCCGAGGTGCACTGGATACGACAAAATATGG-3′
U6-F	5′-TGCGGGTGCTCGCTTCGGCAGC-3′
U6-R	5′ CCAGTGCAGGGTCCGAGGT 3′

### Quantitative real-time PCR

Total RNA was extracted using Trizol solution (Invitrogen, USA) according to the manufacturer’s protocol, and RNAse-free DNase was used to remove DNA contamination. Total RNA concentration and quantity were assessed using a DNA/Protein Analyzer (GeneQuant pro RNA/DNA). cDNA was synthesized from RNA, using a PrimeScript™ RT reagent Kit (TaKaRa). The special primer was used to synthesize miR-302b cDNA, which is shown in Table 1. The cDNA specimens were amplified using an SYBR Premix Ex Taq™ II (TaKaRa). The polymerase chain reaction (PCR) primers used are shown in Table 1. PCR amplification was performed on the IQ5 Optical System real-time PCR machine. β-actin and U6 were used to normalize mRNA and miRNA respectively. Relative quantification of mRNA expression levels was determined using the relative standard curve method according to the manufacturer’s instructions (Bio-Rad).

### MTT assay

The cells were seeded into 96-well plates at a density of 1 × 10^5^ cells/well with 100 uL of 1640, supplemented with 10% fetal bovine serum without antibiotics for 24 h. Thereafter, 0.2 ug of the miR-302b ctrl (empty vector), miR-302b expression vector, siEGFR or siRNA-ctrl oligonucleotide in 25 μl of 1640 and 0.5 μl of lipofectamine 2000 (Invitrogen, USA) in 25 μl of 1640 were preincubated for 5 min at room temperature, respectively, and then mixed together and incubated for additional 25 min at room temperature. After the addition of 50 μl of 1640, the entire mixture was added to the well, and the cells were further cultivated for an additional 1–3 days. Cell viability was assessed using the 3-(4, 5-dimethyl-2-thiazolyl)-2,5-diphenyl-2H-tetrazolium bromide (MTT) assay on FLUOstar OPTIMA (BMG). Each experiment contained three replicates and was repeated at least twice. The data were summarized as mean ± s.d.

### Western blot

The culture of SMMC-7721 cells and the transfection of miR-302b expression vector, miR-ctrl, siEGFR, and siRNA-ctrl were performed as above. All RNA transfections were performed at a final concentration of 100 nM unless otherwise indicated. SMMC-7721 cells were lysed using RIPA buffer, supplemented with protease inhibitor (invitrogen). Protein concentration was estimated by quantitative analyzer (GeneQuant pro RNA/DNA). Protein was then separated with a 8% to 10% SDS-PAGE (Invitrogen), transferred to a nitrocellulose membrane, incubated with the EGFR, pAKT2, AKT2, CCND1, CDK2, p27, and β-actin antibodies (Bioworld, diluted 1/500). After washed three times with TBST, the membrane was incubated with a goat anti-rabbit antibody (Bioworld, diluted 1/5000). Relative protein expression was then normalized to β-actin levels in each sample.

### Immunofluorescence microscopy

To determine the effect of miR-302b/siEGFR on cell proliferation, we also performed immunofluorescence staining using the Ki-67 antibody (Millipore, diluted 1/100). Plasmid miR-302b or siEGFR was transfected into SMMC-7721 cells using Lipofectamine 2000 (Invitrogen Co., Carlsbad, CA, USA) into SMMC-7721 cells, miR-ctrl and siRNA-ctrl as respective controls. After 48 h, transfected SMMC-7721 cells were fixed with 4% formaldehyde for 20 min, then incubated with 0.5% Triton X-100. Anti-Ki-67 antibody (Bioworld, 1:100) was used for immunofluorescence staining. After washed three times with PBS, the cells were incubated with a goat anti-mouse antibody (Millipore, diluted 1:500), and measured by immunofluorescence microscopy.

### Dual luciferase assay

PmirGLO-EGFR-3′UTR-wt vector or pmirGLO-EGFR-3′UTR-mut vector were co-transfected with miR-302b or miR-ctrl into SMMC-7721 cells using lipofectamine 2000 (Invitrogen). Then, reporter gene assays were performed 24 h and 48 h post-transfection using the Dual luciferase Reporter assay system (Promega) according to the manufacturer’s protocol. The normalized firefly luciferase activity was obtained by firefly luciferase activity/Renilla luciferase activity. All experiments were performed at least three times.

### Colony assay

Post-transfected SMMC-7721 cells were resuspended and seeded onto 12-well plates at a density of 2000 cells/well, incubated two weeks later, and then were stained with 0.5% crystal violet for 30 min. Excess dye was rinsed off twice with PBS. The pictures were obtained by using computer software (Bio-Rad quantity one).

### Cell cycle analysis

The SMMC-7721 cells were transfected with miR-302b re-expression vector, miR-ctrl, siEGFR or siRNA*-*ctrl. Cells were harvested by trypsinization, and 1 × 10^6^ cells were used for analysis after 24 h, 48 h, and 72 h. The cells were washed in PBS and fixed in ice-cold ethanol overnight at 4°C. The cells were then washed in PBS and incubated in 1 ml staining solution (20 ug/ml propidium iodide and 10 U/ml RNaseA) for 30 min at room temperature. Cell cycle distributions were assayed by fluorescence-activated cell sorting using a flow cytometer (FACSort; Becton).

### Statistical analysis

Each experiment was repeated at least three times. Numerical data were presented as mean ± s.d.. Unless indicated, the differences between the two groups were analyzed using a Student’s *t*-test (two-tailed). All statistical analyses were performed using SPSS13.0 software (SPSS, Chicago, IL, USA). The linear correlation coefficient (Pearson’s r) was calculated to estimate the correlation between miR-302b values and EGFR levels in the matched HCC tumor specimens.

## Results

### MiR-302b is low-expressed and EGFR is high-expressed in HCC tissue samples and HCC cells

To validate the tumor suppressor role of miR-302b in clinical hepatoma, we analyzed the expression of miR-302b in 27 pairs of clinical HCCs and adjacent nontumorous liver tissues using quantitative real-time PCR (qRT–PCR) and normalized to an endogenous control (U6 RNA). Among the 27 pairs of clinical tissues, down-regulation of miR-302b was observed in 22 (81%) HCC samples compared with their adjacent nontumorous liver tissues, whereas up-regulation of EGFR at mRNA level was found in 21 (78%) HCC tissues compared with adjacent nontumorous counterparts (Figure 1A and B). Moreover, we found that miR-302b was down-regulated in examined HCC cells compared with normal hepatocytes (HL-7702 cells) (Figure 1C). Furthermore, the protein levels of EGFR were up-regulated in four paired tissues (Figure 1D) and in four hepatoma cells compared with adjacent nontumorous liver tissues and normal hepatic cells (Figure 1E). The results suggested that the reduced miR-302b expression and increased EGFR expression were frequent events in human HCC tissues.

**Figure 1:** **Dysregulated miR-302b/EGFR in hepatocarcinoma tissues and cells. A-** qRT–PCR analysis of miR-302b expression in 27 paired HCC tissues and their corresponding adjacent nontumorous livers. The expression of miR-302b was normalized to U6 snRNA. The data are reported as mean ± s.d. (*P < 0.05, Student’s *t*-test). **B-** qRT–PCR analysis of EGFR expression in 27 paired primary HCC tissues and their corresponding adjacent nontumorous liver tissues. The expression of EGFR was normalized to β-actin (*P < 0.05, Student’s *t*-test). **C-** qRT–PCR analysis of miR-302b expression in normal hepatocytes (HL-7702 cells) and HCC cells (Bel7402, Hep3B, HepG2, SMMC-7721 cells), (**P < 0.01, *P < 0.05, Student’s *t*-test). **D-** Western blot analysis of EGFR expression in four pairs of HCC tissues and their corresponding nontumorous liver tissues, with β-actin as an internal control. The intensity for each band was quantified. The value under each lane indicates the EGFR expression in four tumor tissues compared with their corresponding nontumorous liver tissues. **E-** Western blot analysis of EGFR expression in hepatocytes, and hepatoma cells, with β-actin as an internal control. The value under each lane is represented the intensity ratio between hepatoma cells and hepatocytes.

### MiR-302b targets at EGFR

We searched for miR-302b target genes using three computer-aided miRNA target prediction programs, RegRNA, DIANA and TargetScan. As shown in Figure 2A, there is a miR-302b-binding site at 4259-4284nt of the EGFR 3′ UTR. Comparing the human sequence with interspecies homology, we found that the miR-302b targeting sequence was highly conserved among different species. To determine whether EGFR was a direct target of miR-302b, we constructed pmirGLO-EGFR-3′UTR-wt and pmirGLO-EGFR-3′UTR-mut. Later, we have co-transfected miR-302b or miR-ctrl with pmirGLO-EGFR-3′UTR-wt or pmirGLO-EGFR-3′UTR-mut into SMMC-7721 cells. The results showed that miR-302b obviously suppressed the firefly luciferase activity of pmirGLO-EGFR-3′UTR-wt at 24 and 48 h, compared with miR-ctrl (Figure 2B). In addition, we proved that the re-expression of miR-302b did not affect the mRNA expression of EGFR (P > 0.05), but could suppress EGFR at the protein level (50%). Meanwhile, after transfected miR-302b inhibitor into SMMC-7721 cells, the expression of EGFR at mRNA levels did not change. However, transfection of miR-302b inhibitor can increase the expression of EGFR at protein level (Figure 2C), suggesting that miR302b inhibit EGFR expression at translational level but not transcription level in SMMC-7721 cells. Interestingly, as shown in Figure 2D, miR-302b expression level in vivo was inversely-correlated with EGFR mRNA expression level, which was verified by Pearson’s correlation coefficient test, suggesting that miR-302b may relate to EGFR mRNA expression level. Taken together, our data demonstrated that miR-302b targeted at EFGR and suppressed its expression at translation level in SMMC-7721 cells.

**Figure 2:** **MiR-302b targets at EGFR. A**- miR-302b-binding site at 4259–4284 nt of the EGFR 3′ UTR is predicted to be evolutionarily conserved across different species. **B**- 24 and 48 h after transfection, luciferase assay in SMMC-7721 cells. 25-bp regions (wt) miR-302b binding sites in the EGFR 3′ UTR was cloned into pmirGLO Dual-Luciferase miRNA Target Expression vector. Identical constructs mutation was generated. Either miR-ctrl or miR-302b was co-transfected with pmirGLO-EGFR-3′ UTR-wt or pmirGLO-EGFR-3′ UTR–mut into SMMC-7721 cells and luciferase activity assayed after 24 h and 48 h. The normalized firefly luciferase activity was obtained by firefly luciferase activity/Renilla luciferase activity. Luciferase activity of reporter gene (EGFR 3′ UTR-wt) displayed a significant decrease by transfecting miR-302b. These experiments were performed in triplicate, and the results are shown as the mean ± s.d. (**P < 0.01 Student’s *t*-test). **C**- EGFR mRNA and protein expression levels measured by qRT-PCR and western blot 48 h after transfecting with miR-ctrl, miR-302b, inhibitor-ctrl or miR-302b-inhibitor. The intensity for each band was quantified. The value under each lane indicates the expression level of EGFR, which is represented by the intensity ratio between miR-302b or inhibitor and miR-ctrl or inhibitor-ctrl groups. **D**- Inverse correlation between miR-302b and EGFR expression in HCC tissues. Expression of EGFR analyzed by qRT–PCR and normalized to β-actin. The miR-302b expression was examined by qRT–PCR analysis and normalized to U6 expression. Statistical analysis was performed using Pearson’s correlation coefficient (r = −0.48, *P < 0.05).

### The miR-302b inhibited the growth of SMMC-7721 cells through targeting EGFR

To examine the effects of miR-302b on the growth of SMMC-7721 cells through targeting EGFR, we designed the siRNA for EGFR (siEGFR), which induced 50% decrease of EGFR expression both at the mRNA and protein levels in SMMC-7721 cells. At the same time, we transfected miR-302b into SMMC-7721 cells and observed a thirty-fold increase of the miR-302b expression (Figure 3A). MTT assay showed that miR-302b overexpression resulted in the suppression of the SMMC-7721cells growth at 48 and 72 h, which was in accord with the effect of siEGFR (Figure 3B). To further examine the inhibitory role of miR-302b and siEGFR in SMMC-7721 cells, colony formation assay was employed. Notably, miR-302b/siEGFR–transfected cells displayed fewer and smaller colonies compared with their respective controls (Figure 3C). Moreover, miR-302b and siEGFR suppressed cell proliferation at the G0/G1 phase at 24 h, 48 h and 72 h time points (Figure 3D). Finally, to determine the growth fraction of HCC cells after overexpression of miR-302b/siEGFR, we performed Ki-67 immunofluorescence staining. The signal of Ki-67 in the miR-302b/siEGFR–transfected SMMC-7721 cells was visibly low compared with that of the cells transfected with their respective controls (Figure 3E). These findings demonstrated that the effect of miR-302b re-expression on cell proliferation was consistent with that of siEGFR on SMMC-7721 cells, suggesting that miR-302b may inhibit the growth of SMMC-7721 cells through targeting EGFR.

**Figure 3:** **Overexpression of miR-302b and knockdown of miR-302b-target gene EGFR decrease hepatoma cell growth and induce G1/S arrest in vitro. A**- qRT-PCR analysis of miR-302b in SMMC-7721 cells transfected with miR-302b over-expression construct and miR-ctrl (left). qRT–PCR (upper portion) and western blot analysis (lower portion) were performed to determine the expression level of EGFR after transfection of siEGFR and siRNA-ctrl. (*P < 0.05, **P < 0.01, Student’s *t*-test) (right). **B**- The effects of miR-302b or siEGFR on SMMC-7721 cell proliferation were determined by MTT assay at 24 h, 48 h, and 72 h after transfecting of miR-302b over-expression construct or siEGFR, with miR-ctrl or siRNA-ctrl as the respective controls (*P < 0.05, **P <0.01, Student’s *t*-test). **C**- Representative results of colony formation of SMMC-7721 after transfection of miR-302b re-expression or siEGFR. **D**- Cell cycles determined in SMMC-7721 cells after transfection of miR-302b over-expression construct or siEGFR at 24 h, 48 h, 72 h, with miR-ctrl or siRNA-ctrl as the respective controls. Histogram indicates the percentage of cells at G0–G1, S, and G2–M cell-cycle phases (*P < 0.05, Student’s *t*-test). **E**- Expression of Ki-67 was verified by immunofluorescence staining after transfecting with miR-ctrl, miR-302b, siRNA-ctrl, or siEGFR. Merged pictures are overlays of both Ki-67 red signals and nuclear staining by DAPI (blue).

### MiR-302b inhibits cell proliferation through EGFR*-*dependent cell cycle regulation

AKT is the key molecule in the signaling pathway, which is regulated by EGFR*.* Abnormal expression of EGFR leads to a change of AKT expression [19,20]*.* The re-expression of miR-302b reduced the expression of AKT2, pAKT2, and its downstream gene CCND1, CDK2, and up-regulated CDK inhibitor p27 in SMMC-7721 cells (Figure 4A). Similar results were proved by the treatment of siEGFR (Figure 4B), suggesting that miR-302b may suppress the growth of SMMC-7721 cells by targeting the EGFR/AKT2/CCND1 signaling pathway.

**Figure 4:** **MiR-302b inhibits cell proliferation through EGFR-dependent cell cycle regulation. A**- Western blot results of miR-302b-targeted EGFR and non-direct targeted cell cycle regulation proteins in SMMC-7721 cells after transfection of miR-302b over-expression construct and miR-ctrl. β-actin was used as an internal control. **B**- Protein level of EGFR and relative cell cycle regulation proteins were measured by western blot 48 h after transfection of siEGFR and siRNA-ctrl into SMMC-7721 cells. The expression of the proliferation-related gene was normalized to β-actin. The intensity for each band was quantified. The value under each lane indicates the relative expression level of the proliferation-related gene, which is represented by the intensity ratio between miR-302b and miR-ctrl or inhibitor and inhibitor-ctrl groups.

## Discussion

HCC is a primary lethal neoplasm of the liver and the third cause of cancer-related deaths worldwide [21]. However, its underlying molecular mechanism remains largely unknown. In the past ten years, microRNAs (miRNAs) have been found to be involved in the initiation and progression of HCC. According to its tumorigenesis function, miRNAs can be divided in two classes:oncogenes and tumor suppressor genes [22]. Many oncogenic miRNAs, such as miR-221 and miR-222, are involved in sustaining proliferative signaling, resisting growth suppression and apoptosis, enabling immortality, prompting angiogenesis, invasion and metastasis, evading and so on [23-28], whereas tumor suppressor miRNAs are involved in the reverse processes. Let-7 family and miR-101, as potential tumor suppressors, were markedly decreased in HCC cells [29,30]. Recent studies proved that the miR-302-367 cluster is down-regulated in cervical cancer cells and gastric adenocarcinoma [31,32]. Our study showed that the expression of the miR-302b was frequently down-regulated in clinical HCC tissues and in SMMC-7721 cells (Figure 1). Thus, we supposed that miR-302b might be a novel tumor-suppressor miRNA.

Human epidermal growth factor receptor (EGFR/HER/ErbB) family of tyrosine kinases plays a major role in the etiology and progression of many carcinomas, including HCC. Increased expression of EGFR/HER1 occurs frequently in different human tumor types, and is involved in the early stages of human hepatocarcinogenesis [33,34]. In our study, increased expression of EGFR was observed in the HCC samples and HCC cells (Figure 1D and E). Over-expression of EGFR is also related to the gene amplification of EGFR and deficiency of EGFR targeting miRNA. There seemed to be a negative correlation between the expression of EGFR and that of miR-302b in HCC tissues (Figure 1A and B), implying that EGFR might be a novel target of miR-302b. Further bio-information analysis showed that there was a miR-302b-binding site at 4259–4284 nt of the EGFR 3′ UTR. The dual-luciferase reporter assays demonstrated that miR-302b targeted directly to EGFR through the suppression of translation (Figure 2B). In this research, we examine the relationship between miR-302b and EGFR at both of the transcription level and translational level, in which miR-302b was verified to silence EGFR at translational level from in vitro and in vivo clinical samples. At the transcription level, we tested relationship between miR-302b and EGFR by using Pearson’s correlation coefficient test in 27 paired HCC tissues and found that they have inverse correlation in mRNA level (Figure 2D). Whereas in SMMC-7721 cell lines, the correlation between miR-302b and EGFR didn’t show significant difference (Figure 2C), but it exhibited the correlation trend, which were consistent with the results of that in HCC tissues.

EGFR induces activation of the Ras/Raf/MEK/MAPK pathway through either Grb2 or Shc adaptor proteins, and that of PI3K/AKT/CCND1 pathway by recruitment of the p85 regulatory subunit to the activated receptors [35]. The activation of EGFR/AKT/NF-kB/CCND1 survival signaling pathway has been certified in cholesteatoma epithelium [36]. Function of dominant negative EGFR shows that dominant negative EGFR induces G0/G1 arrest by decreasing the expression of phosphorylated retinoblastoma protein, phosphorylated GSK-3β, CCND1, and by increasing expression of p21 and p27 in human gastric cancer cells SGC-7901 and NCI-N87 [37]. AKT2 is essential for progressing from the G0/G1 to the S-phase by activating the positive regulator of G1/S transition, including CCND1, CCND2, and CCNE1, during cell cycle progression [38]. CCND1, as a AKT2 downstream gene, is expressed in the G1 phase of the cell cycle, together with its CDK partner, CDK2. p27, as a CDK inhibitor, could be combined with CCND1-CDK2 complex to restrain CDK2 activity [39]. Our results showed that miR-302b may inhibit the growth of SMMC-7721 cells through targeting EGFR, and that the cell cycle progression was arrested at the G0/G1-phase (Figure 3). At the same time, the expression of AKT2 was down-regulated, and CCND1 and CDK2 were reduced by miR-302b, while the expression of CDK inhibitor p27 was up-regulated (Figure 4). A few of the miR-302b targets have been found, including AKT1, CCNA, CDK2, CCND1/D2, and BMI-1 [40]. These genes are involved in the regulation of the cell cycle. In order to prove the biological effects of miR-302b on inhibition of EGFR, siEGFR was used. The results showed that the effect of miR-302b re-expression on the cell proliferation was consistent with that of siEGFR in SMMC-7721cells, suggesting that miR-302b may suppress the growth of SMMC-7721 cells by targeting the EGFR/AKT2/CCND1 signaling pathway.

## Conclusions

In conclusion, the dysregulation of miR-302b is a frequent event in human hepatocarcinoma. The high-expression of EGFR is related to the down-regulation of miR-302b in HCC. The re-expression of miR-302b suppresses the growth of hepatoma cells may due to targeting the EGFR/AKT2/CCND1 pathway, suggesting that miR-302b may be an effector in gene therapy of HCC.

## Competing interests

The authors declare that they have no competing interests.

## Authors’ contributions

CH and JYY developed the hypotheses. LMW and LLH executed the experiments. JYY, TSS and ZFL provided the experimental facilities and research funds. LMW, JYY, XS, and CH wrote and revised the paper. All authors read and approved the final manuscript.

## Pre-publication history

The pre-publication history for this paper can be accessed here:

http://www.biomedcentral.com/1471-2407/13/448/prepub
